The article "Do precarious female employment and political autonomy affect the under-5 mortality rate? Evidence from 166 countries" was retracted in 2024. Reasons: original data or images not available; unreliable results or conclusions; concerns about the data; concerns about the results or conclusions.

# Do precarious female employment and political autonomy affect the under-5 mortality rate? Evidence from 166 countries

**DOI:** 10.1371/journal.pone.0269575

**Published:** 2022-06-27

**Authors:** Sasmoko, Shabnam, Wiwik Handayani, Abdelmohsen A. Nassani, Mohamed Haffar, Khalid Zaman

**Affiliations:** 1 Primary Teacher Education Department, Faculty of Humanities, Bina Nusantara University, Jakarta, Indonesia; 2 Department of Humanities and Social Sciences, National Institute of Technology (NIT) Kurukshetra, Haryana, India; 3 Faculty of Business and Economics, Universitas Pembangunan Nasional (UPN), Veteran Jawa Timur, Indonesia; 4 Department of Management, College of Business Administration, King Saud University, Riyadh, Saudi Arabia; 5 Department of Management, Birmingham Business School, University of Birmingham, Birmingham, United Kingdom; 6 Department of Economics, The University of Haripur, Khyber Pakhtunkhwa, Haripur, Pakistan; University of Almería, SPAIN

## Abstract

The United Nations’ Sustainable Development Goals (SDGs) were designed to benefit the globalized world by safeguarding economic and environmental resources necessary for quality health and well-being and moderate growth and development. The study focused specifically on SDG-3 (good health and well-being), SDG-5 (gender equality), and SDG-8 (decent work and economic growth) to identify the most significant influencing factors that can affect the under-5 mortality rate in a large cross-section of 166 countries. The research used three different regression apparatuses to produce consistent and unbiased estimates: cross-sectional, robust least squares, and quantile regression approaches. Additionally, the innovation accounting matrix technique examines the intertemporal relationships between the variables over the time horizon. The data reveal that precarious female employment increases the under-5 mortality rate. On the other hand, women’s political autonomy continued economic growth, and higher immunization coverage is supporting factors for achieving healthcare sustainability agenda. The ex-ante analysis indicates that per capita income will significantly impact the under-5 mortality rate, followed by women’s political autonomy, insecure female employment, and immunization coverage during the next ten years. The results are consistent with other health indicators such as the health damage function, labour market function, and wealth function. The study suggests that the more unlocking women’s potential in political life, the more likely it is to achieve equitable healthcare choices and reduce the mortality rate among children under five. As a result, there is an urgent need for women to have an equitable share of the labour market to appropriately meet their family healthcare demands.

The article "Do precarious female employment and political autonomy affect the under-5 mortality rate? Evidence from 166 countries" was retracted in 2024. Reasons: original data or images not available; unreliable results or conclusions; concerns about the data; concerns about the results or conclusions.

## 1. Introduction

The United Nations’ Sustainable Development Goals (SDGs) are designed to move the world closer to prosperity. The SDGs 3, 5, and 8 were reviewed in this research, which analysed data from a broad cross-section of nations to determine the likely reasons for under-5 mortality when a country faces an unanticipated labour supply shock, especially among women. Additionally, gender inequality and the economic crisis were examined. SDG-3’s primary objective is to guarantee healthy lifestyles for all people by reducing global maternal mortality and under-five mortality ratios. The stated objective is tied to SDG-5, highlighting the need to empower women and girls in both the public and private spheres. The stated objective underlines the critical nature of ensuring equal access to universal healthcare benefits for women participating in economic and political concerns. The SDG-8 underlined the need to achieve a higher economic output via technological innovation and variety [1]. Given the importance of the stated objectives, the current research used the declared holistic objectives to modify economic and healthcare policies to guarantee that people live healthy and affluent lives due to labour market changes.

In many areas of the globalised world, vulnerable female employment has exceeded 90%, leading to an increased under-5 mortality rate (more than 100 per 1,000 live births) and a reduced women’s autonomy index score of as little as one-quarter of the index value. Female vulnerability is more widespread in various situations, resulting in a greater infant mortality rate and reduced women’s autonomy in many contexts. On the other hand, countries with a higher female labour force participation rate and more economic equality diminish vulnerable female employment, resulting in a lower under-5 death rate and a higher Women’s Autonomy Index score. The low vaccination rate poses a threat to the under-5 mortality rate. Table 1 summarizes the facts by offering a few glimpses of them.

**Table 1:** A few facts about socio-economic sufferings leading to under-5 mortality rates.

Countries	Female Vulnerable Employment (% of female employment)	Under-5 Mortality Rate (Per 1,000 live births)	Women Business and the Law Index Score (Scale 1 to 100)	Measles Immunization Rate (% of children ages 12–23 months)
Afghanistan	89.47	60.3	38.125	64
Congo, Rep.	90.70	47.8	49.375	73
Equatorial Guinea	79.61	81.8	51.875	53
Guinea-Bissau	80.31	78.5	42.500	79
Haiti	81.27	62.8	63.75	65
India	75.28	34.3	74.35	95
Indonesia	57.08	23.9	64.375	88
Mauritania	75.67	72.9	48.125	78
Niger	97.97	80.4	59.375	79
Nigeria	85.21	117.2	63.125	54
Pakistan	70.16	67.2	52.501	81
Papua New Guinea	84.01	44.8	60	37
Sierra Leone	92.94	109.2	63.125	93

Source: World Bank [2].

The article "Do precarious female employment and political autonomy affect the under-5 mortality rate? Evidence from 166 countries" was retracted in 2024. Reasons: original data or images not available; unreliable results or conclusions; concerns about the data; concerns about the results or conclusions.

The study is limited to a few variables affecting the healthcare sustainability agenda, including vulnerable female employment, under-5 mortality, immunization coverage, and women’s political autonomy. Due to a lack of direct evidence, the authors believe that when these factors are combined, they result in a significant policy gap for preventing under-5 mortality in various countries worldwide. Adeleye et al. [3] examined the insecure nature of female employment in India and its impact on its economic growth. They identified a negative correlation between the two investigated factors. As a result, it was established that vulnerable female employment had a detrimental effect on the country’s economic growth. Significant adjustments must be made to the female workforce in order for it to narrow the gender divide and participate in economic and political concerns. Women’s increased vulnerability to violence in agriculture may be addressed by encouraging them to engage in industrial and service industries, which will improve their living conditions. Akkan and Serim [4] observed that Turkish women were confronted with unprecedented working challenges. Numerous factors contribute to such poor healthcare outcomes, including family life problems, a tight labour market structure, gender gaps in education, inflexible employment laws, a lack of childcare facilities, and ineffective work policies. These influences reduce women’s autonomy, precipitating a severe economic crisis that exacerbates social differences by establishing class disparities. Gammage et al. [5] emphasized the need to pursue feminist changes to improve one’s life and contribute to society. It may be accomplished by establishing universal healthcare coverage, establishing a social safety net, and implementing social labour market adjustments through the decent programme. Kashyap and Behrman [6] examined the various causes of India’s high female under-5 death rate, concluding that the primary cause is a lack of parental healthcare investment in the female child, resulting in poor health. If a country wants to minimize female under-5 mortality rates, it must shift the traditional parental perspective toward giving equal importance to their children. Shajan and Sumalatha [7] examined the possible association between a mother’s profession and her children’s health in Indian youngsters. They identified other startling facts, such as working mothers’ inability to provide their children with their undivided attention, which results in their bad health. On the other side, mothers who remain at home with their children and are unemployed may give their children more healthy time, which helps them improve their health. Additionally, working women with better jobs and higher-quality skills were better able to manage their children’s healthcare status than working moms who remained in the subsistence sector and struggled to pay household expenses. As a consequence, the infant is malnourished and ill. Investing in women to ensure they have an equitable education and develop their technical abilities will benefit their ability to care for their families and children efficiently. Hossain et al. [8] discovered that educated mothers, affluent families, and children who receive parental care have a lower incidence of under-5 malnutrition in their children in Bangladesh than mothers who are less educated, come from low-income families, and lack access to adequate healthcare coverage. Daher-Nashif and Bawadi [9] stressed the need for equitable healthcare access to reduce maternal mortality and contribute to the attainment of global sustainable development goals. Balaj et al. [10] revealed significant correlations between parental education and a reduction in child mortality. The data imply that the more educated women there are compared to males, the higher the possibility of lowering child mortality. This demonstrates sound analytical judgment in ensuring and investing in the education and health of women in order to assist their families and children. Abreha and Zereyesus [11] stated that women’s equality in family decision-making significantly improves children’s health outcomes, enabling sub-Saharan African nations to advance in their goal of political autonomy. Abreha et al. [12] argued that women’s equality and empowerment are critical for achieving equitable educational opportunities in Ethiopia. They empower women to become more information-oriented, enabling them to promote family saving to reduce their child’s undernutrition, prevent it from contracting pneumonia, and prevent becoming anemic. The research stressed the need for increased investment in women’s education, which would result in greater empowerment of women in all aspects of public and private life. Numerous research undertaken in Sub-Saharan African countries, notably Yaya et al. [13] have proven a statistically significant positive link between numerous aspects of women’s empowerment and improved child healthcare and nutritional status. To improve children’s health and nutrition, policies and initiatives should prioritize women’s economic and familial autonomy since this is likely to result in more positive healthcare changes across countries. According to Panday et al. [14], boosting women’s status would positively affect their children’s welfare, resulting in better sustainable healthcare results. Bhowmik et al. [15] uncovered critical evidence about women’s education and its impact on reducing socio-economic externalities. Women who obtained any education, from elementary to higher school, were less likely to marry before 18 than women who had no education. Additionally, women with a secondary or higher education are less likely to become adolescent moms than women without a secondary or higher education. Finally, pre-marital relationships before the age of eighteen and mothers of teens who are unable to complete their education. Thus, the need for women and girls to be empowered via technical and compulsory education, which has the potential to minimize negative social externalities, becomes even more pressing. The study proposed the following research hypotheses based on the literature review:

H1: It is projected that vulnerable female employment would raise the mortality rate of children under the age of five.

The article "Do precarious female employment and political autonomy affect the under-5 mortality rate? Evidence from 166 countries" was retracted in 2024. Reasons: original data or images not available; unreliable results or conclusions; concerns about the data; concerns about the results or conclusions.

H2: Women’s autonomy is expected to decrease suffering in healthcare and reduce the under-5 mortality rate.

H3: Continued economic growth benefits healthcare spending, leading to decreased healthcare damage across countries; and

H4: Increased vaccination rates are anticipated to result in a drop in under-5 mortality.

The study adds by proposing a healthcare model in which vulnerable female employment, women’s political autonomy, immunization coverage, and a country’s per capita income all affect the under-5 mortality rate. Earlier studies mostly ignored precarious female work when developing models that lacked economic strategies to reduce under-5 mortality [16–18]. Precarious female employment has been extensively studied previously in terms of a variety of socio-economic factors, including education disparities between formal and informal education [19], labour market rigidities [20], family formation [21], health consequences [22], labour market shocks associated with refugee inflows [23], and social norms [24]. However, little or no progress has been made regarding women’s engagement in managing political affairs in connection to insecure female labour and under-5 mortality rates. Continuous economic progress resulted in a beneficial decrease in the mortality rate of children under the age of five, as defined by the United Nations’ sustainable development goal-8 (decent employment and economic growth). In light of the study’s contribution, the following research objectives are proposed:

- To analyze the influence of precarious female employment on the under-5 mortality rate within the framework of the decent work agenda.
- To assess the role of women in managing political affairs in reducing under-5 mortality, and iii) To understand the need to improve a country’s per capita income and vaccination rate efficiently to solve child health concerns.

The article "Do precarious female employment and political autonomy affect the under-5 mortality rate? Evidence from 166 countries" was retracted in 2024. Reasons: original data or images not available; unreliable results or conclusions; concerns about the data; concerns about the results or conclusions.

These objectives have been set to ascertain the critical factors affecting the under-5 mortality rate among countries.

## 2. Data and methodology

The study estimated vulnerable female employment (as a percentage of total female employment) (referred to as FVE), under-5 mortality rate (per 1,000 live births) (referred to as U5MR), women business and law index score (a proxy for women’s political autonomy) (referred to as WPA) (scale 1–100), and GDP per capita (constant 2010 US dollars) (denoted by GDPPC). The U5MR examined the United Nations’ SDG-3 on health and well-being; SDG-5 on gender equality; and SDG-8 on decent work on economic development and vulnerable female employment. Immunization against measles (percent of children aged 12–23 months) (designated by IMUN) is utilized as the study’s control variable since low immunization rates raise U5MR across nations.

The research examined the effect of numerous variables on the death rate of children under the age of five. The innovative and substantial addition to the literature is the use of vulnerable female employment as a predictor of under-five mortality. Based on cross-sectional data gathered from 166 nations at a particular time, i.e., 2019, and the reality that insecure female labour is increasing internationally, resulting in adverse health consequences, a greater incidence of under-5 mortality, and lower women’s political autonomy. Additionally, poor vaccination rates harmed governments’ efforts to achieve a sustainable healthcare agenda. The data comes from the World Bank’s World Development Indicators [2]. The cross-sectional study design enables collecting data from a varied range of countries on the specified factors that influenced under-5 mortality rates at a specific time. The study aims to gather and evaluate essential data on recent changes in under-five mortality rates across a large cross-section of nations. It permits the research to conduct two independent analyses of the connections between variables. First, an analytical cross-sectional investigation is conducted. The research aims to explain how and why under-5 death rates are increasing due to rising female vulnerable work, poor economic development, low vaccination rates, and growing gender disparity. On the other hand, descriptive statistics were used to characterize the aforementioned issues. Cross-sectional studies allow for collecting data from a large number of countries and the comparison of group differences. Over time, longitudinal studies collect data from various countries, often focusing on a small number of countries with comparable characteristics. Furthermore, cross-sectional dependence occurs in most instances in the panel data, resulting in skewed and inconsistent parameter estimations if the issue is not handled effectively. The study’s scope is confined to examining the recent trend in under-5 death rates across nations at specified periods rather than examining the variables’ long- and short-run associations. Consequently, the study employs cross-sectional analysis to derive an answer from previously collected data.

The article "Do precarious female employment and political autonomy affect the under-5 mortality rate? Evidence from 166 countries" was retracted in 2024. Reasons: original data or images not available; unreliable results or conclusions; concerns about the data; concerns about the results or conclusions.

For this research, the year 2019 was selected for various reasons. It was chosen because the United Nations Millennium Development Goal-4, which sought to halve global child mortality by 2015, had not been met in many regions of the globalized globe. Additionally, it was tied to the United Nations Sustainable Development Goal-3, which fulfilled objectives for lowering child mortality to the desired level using the given measure. Consequently, the study assessed recent progress in lowering under-5 mortality rates across countries.

The research assessed three theoretical viewpoints in order to understand better the potential causes of negative healthcare externalities across countries, namely:

**i) Health Damage Function:** The Function identifies various factors that have a detrimental effect on long-term healthcare outcomes, including a lack of healthcare infrastructure, illiteracy, lower school enrollment, direct exposure to pollution, a lack of sanitation facilities, and a lack of institutional-based interventions [25]. Additionally, it highlights low-income family income [26], inherited congenital disorders, and a dearth of institutional-based solutions [27]. Globally, infant mortality rates are predicted to drop due to increasing investment in healthcare infrastructure and improved literacy. By increasing literacy, environmental dangers and sanitation problems may be avoided, decreasing under-5 death rates. Fig 1 illustrates a possible strategy for lowering unfavourable health outcomes in the community.

**Fig 1:** Healthy interventions to reduce under-5 mortality rates. Source: Adapted from Pillai& Christina [28] and authors extract.

**ii) Labor Market Function**: Supply and demand shock primarily affect the labour market function. As a consequence of labour market shocks, wage disparities and gender inequality have increased. Women’s potential was repressed, and little investment in the female labour force resulted in a severely disadvantaged female labour force. Precarious female labour undermines the United Nations’ aim of gender parity, decreasing women’s healthcare outcomes [29–31]. Fair and equitable labour market adjustments would aid in the road toward equal work possibilities and a similar wage structure around the world. Fig 2 illustrates the remedial measures that may improve the fairness of labour force changes.

The article "Do precarious female employment and political autonomy affect the under-5 mortality rate? Evidence from 166 countries" was retracted in 2024. Reasons: original data or images not available; unreliable results or conclusions; concerns about the data; concerns about the results or conclusions.

**Fig 2:** Equitable labor market reforms. Source: Adapted from Vives et al. [29] and authors extract.

**iii) Wealth Function:** This function is mainly responsible for increasing per capita income, increasing job opportunities, and improving the nation’s healthcare system. Increased per capita income is being utilised to invest in socio-economic infrastructure and gender equality measures to assist women in entering the workforce [32–34]. To achieve more favourable healthcare outcomes, it is necessary to have a healthy workforce and execute institutional intervention programmes to reduce under-5 mortality. For convenience, Fig 3 depicts the wealth function.

**Fig 3:** Wealth function. Source: Adapted from Mujeed et al. [33] and authors extract.

Based on the theoretical literature support, the study shows the estimated regression equation, i.e.,

$$\begin{array}{l} \ln(U5MR)=\alpha_{0}+\alpha_{1}\ln(FVE)+\alpha_{2}\ln(WPA)+\alpha_{3}\ln(GDPPC)+\alpha_{4}\ln(IMUN)+\varepsilon \\ ∴\frac{\partial \ln(FVE)}{\partial \ln(U5MR)}>0,\frac{\partial \ln(WPA)}{\partial \ln(U5MR)}<0,\frac{\partial \ln(GDPPC)}{\partial \ln(U5MR)}<0;\frac{\partial \ln(IMUN)}{\partial \ln(U5MR)}>0 \end{array}$$ (1)

Where U5MR shows an under-5 mortality rate, FVE shows vulnerable female employment, WPA shows women’s political autonomy, GDPPC shows GDP per capita, IMUN shows immunization rate, ’ln’ shows natural logarithm, and ε shows error term.

Eq (1) illustrates that vulnerable female employment is predicted to have a detrimental effect on the healthcare sustainability agenda by increasing the mortality rate of children under five. On the other hand, political autonomy for women, a high per capita income, and a low vaccination rate would all reduce under-5 mortality rates across countries. Three feasible econometric procedures were employed to analyse Eq (1): cross-sectional regression methods, robust least squares regression estimator, and quantile regression methods.

The following justifies the usage of the specified regression techniques, i.e., it is feasible to estimate the coefficient at a particular moment in time using cross-sectional regression methods. Diagnostic tests must be performed prior to interpreting the results. The estimated results should have a normally distributed probability, with no signs of autocorrelation or heteroskedasticity. Eq (2) illustrates the cross-sectional regression equation for an estimate, which is referred to as

$$\ln{\left(U5MR\right)}_{i,t}=\alpha_{0}+\alpha_{1}\ln{\left(FVE\right)}_{i,t}+\alpha_{2}\ln{\left(WPA\right)}_{i,t}+\alpha_{3}\ln{\left(GDPPC\right)}_{i,t}+\alpha_{4}\ln{\left(IMUN\right)}_{i,t}+\varepsilon_{i,t}$$ (2)

Where, ‘i’ represents cross-section of 166 countries and ‘t’ shows time period.

The article "Do precarious female employment and political autonomy affect the under-5 mortality rate? Evidence from 166 countries" was retracted in 2024. Reasons: original data or images not available; unreliable results or conclusions; concerns about the data; concerns about the results or conclusions.

Due to the structural breakdowns in the data set, a large residual and leverages value may be noticed in cross-sectional regression; consequently, these values may be reduced by doing the regression analysis using robust least squares regression estimators. The M-estimator [35], the S-estimator [36], or the MM-estimator may be used [37]. The first estimator absorbed the enormous residuals in the dependent variable, enabling the standard deviation of the traditional regression model to be used to build the model. The S-estimator focused on independent variable outliers, which resulted in high leverage values for the dependent variables. Finally, the MM-estimator preserves both the M- and S-estimators, which helps reduce the regression model’s high leverage and residual values. In this method, estimation was carried out utilising the MM-estimator. Eq (3) illustrates the robust least-squares specification, i.e.,

$${\left[\ln{\left(U5MR\right)}_{i,t}\right]}_{MM}=\alpha_{0}+\alpha_{1}{\left[\ln{\left(FVE\right)}_{i,t}\right]}_{MM}+\alpha_{2}{\left[\ln{\left(WPA\right)}_{i,t}\right]}_{MM}+\alpha_{3}{\left[\ln{\left(GDPPC\right)}_{i,t}\right]}_{MM}++\alpha_{4}{\left[\ln{\left(IMUN\right)}_{i,t}\right]}_{MM}+{\left[\varepsilon_{i,t}\right]}_{MM}$$ (3)

Where, MM shows robust least square MM estimator.

Finally, the regression results may diverge into different quantile distributions that cannot be predicted using cross-sectional or other regression techniques, including robust least squares regression. Additionally, both of the aforementioned regression techniques produce mean regression estimates but are unable to produce median regression estimates at the 0.5 quantile distribution; thus, the quantiles regression method is the best fit for the data set to overcome this limitation and produce median regression estimates for the data Eq (4), which illustrates the median regression equation for easy reference, i.e.,

$$\ln{\left(U5MR\right)}_{0.5o}=\tau_{0}+\tau_{1}\ln{\left(FVE\right)}_{0.50}+\tau_{2}\ln{\left(WPA\right)}_{0.50}+\tau_{3}\ln{\left(GDPPC\right)}_{0.50}+\tau_{4}\ln{\left(IMUN\right)}_{0.5}+\varepsilon_{0.50}$$ (4)

Where ‘0.50’ shows the median estimates of the regression model of the respective variables.

The article "Do precarious female employment and political autonomy affect the under-5 mortality rate? Evidence from 166 countries" was retracted in 2024. Reasons: original data or images not available; unreliable results or conclusions; concerns about the data; concerns about the results or conclusions.

To predict the relationship between the stated variables and the regression estimations, the variance decomposition analysis (VDA) was applied. The VDA analysis enables the intertemporal interaction between variables across time and hence provides forecast estimates for observing the changes in provided variables over time. Eq (5) depicts the VDA equation, i.e.

$$\begin{array}{l} Var(\sigma (U5MR,FVE)=Var(E[\sigma ⊥FVE])+E[Var(\sigma ⊥FVE)]\\ \Rightarrow Var(E[\sigma ⊥FVE])\leq Var(\sigma [U5MR,FVE)]\\ Var(\sigma (U5MR,WPA)=Var(E[\sigma ⊥WPA])+E[Var(\sigma ⊥WPA)]\\ \Rightarrow Var(E[\sigma ⊥WPA])\leq Var(\sigma [U5MR,WPA)]\\ Var(\sigma (U5MR,GDPPC)=Var(E[\sigma ⊥GDPPC])+E[Var(\sigma ⊥GDPPC)]\\ \Rightarrow Var(E[\sigma ⊥GDPPC])\leq Var(\sigma [U5MR,GDPPC)]\\ Var(\sigma (U5MR,IMUN)=Var(E[\sigma ⊥IMUN])+E[Var(\sigma ⊥IMUN)]\\ \Rightarrow Var(E[\sigma ⊥IMUN])\leq Var(\sigma [U5MR,IMUN)] \end{array}$$ (5)

Eq (6) depicts the mean sequence error term for the set of variables’ predictors, i.e.

$$\begin{array}{l} MSE_{\mu }=E_{FVE}[MSE_{\mu }(FVE)]\\ MSE_{\mu }=E_{WPA}[MSE_{\mu }(WPA)]\\ MSE_{\mu }=E_{GDPPC}[MSE_{\mu }(GDPPC)]\\ MSE_{\mu }=E_{IMUN}[MSE_{\mu }(IMUN)] \end{array}$$ (6)

Where, MSE shows mean square error term.

## 3. Results and discussion

The variables indicated in Table 2 have descriptive statistics included. Children under the age of five saw a mortality rate of 117.200 deaths per 1,000 live births, with a mean of 27.819 deaths per 1,000 live births. The standard deviation number of 28.030 indicates that the mean value of under-5 mortalities may increase or decrease within the provided deviation value, showing that the variable has significant volatility. The proportion of vulnerable female employment is the highest at 98.770 percent of the entire female population. The lowest and average percentages, by contrast, are 0.040 percent and 39.843 percent, respectively. As stated, the distribution of the aforementioned variable is positively skewed with a high kurtosis value. The measure of women’s political autonomy ranges from 26.250 to 100, with a mean of 75.515 in between. The average per capita income and vaccination rates are US$13,290.58 and 87.198 percent, respectively. Increased female vulnerability and inadequate vaccination rates contribute to an increase in under-5 mortality. In comparison, data indicate that sustained economic growth and women’s political autonomy likely to benefit the global healthcare sustainability agenda.

**Table 2:** Descriptive statistics.

Methods	U5MR	FVE	WPA	GDPPC	IMUN
Mean	27.819	40.258	75.515	13290.58	87.198
Maximum	117.200	98.770	100	111043.5	99
Minimum	2.100	0.040	26.250	208.074	33
Std. Dev.	28.030	30.949	17.577	18825.35	13.910
Skewness	1.323	0.392	-0.892	2.268	-1.774
Kurtosis	3.897	1.709	3.332	8.588	5.921

Note: U5MR shows an under-5 mortality rate, FVE shows female vulnerable employment, WPA shows women’s political autonomy, GDPPC shows GDP per capita, IMUN shows immunization rate.

The article "Do precarious female employment and political autonomy affect the under-5 mortality rate? Evidence from 166 countries" was retracted in 2024. Reasons: original data or images not available; unreliable results or conclusions; concerns about the data; concerns about the results or conclusions.

According to the correlation matrix displayed in Table 3, vulnerable female employment is positively linked with the under-5 mortality rate, with a correlation estimate of 0.833 and a p-value<0.000. On the other hand, both women’s political autonomy and per capita income were negatively linked with the under-5 mortality rate, with correlation magnitudes of -0.327 p<0.000 and -0.486 p<0.000, respectively. The results established that women’s engagement in economic and political life benefits the goal of healthcare sustainability. On the other side, it has been shown that sustained economic expansion reduces under-5 mortality while concurrently boosting national healthcare spending across countries. There is a negative association between vaccination rate and under-5 mortality rate, implying that increasing the vaccination rate reduces the under-5 death rate across nations. Additionally, vaccination rates are favourably connected with sustained economic development and women’s empowerment; hence, it is critical to unleashing women’s economic potential to advance the global health sustainability agenda.

**Table 3:** Correlation matrix.

Variables	U5MR	FVE	WPA	GDPPC	IMUN
U5MR	1				
	-----				
FVE	0.832	1			
	(0.000)	-----			
WPA	-0.327	-0.254	1		
	(0.000)	(0.000)	-----		
GDPPC	-0.486	-0.603	0.353	1	
	(0.000)	(0.000)	0.000)	-----	
IMUN	-0.616	-0.507	0.199	0.305	1
	(0.000)	(0.000)	(0.010)	(0.000)	-----

Note: U5MR shows an under-5 mortality rate, FVE shows female vulnerable employment, WPA shows women’s political autonomy, GDPPC shows GDP per capita, and IMUN shows immunization rate. small bracket shows probability value.

Three types of regression equipment were employed to validate the direction and amplitude of regressors on the regressand (see Table 4). The data indicate that vulnerable female employment has a detrimental effect on reaching the healthcare sustainability target. In all three regression mechanisms analyzed, insecure work tends to raise the mortality rate of children under the age of five. Nonetheless, the influence on the "response variable" is more significant in quantile regression than in other forms of regression, such as cross-sectional and robust least squares regressions. According to the data, unstable female employment is the adverse factor contributing to the increase in the mortality rate of children under the age of five in all countries analysed. Numerous prior studies have shown a negative correlation between vulnerable female employment and the implementation of a sustainable healthcare agenda in several economic situations with various socioeconomic and environmental characteristics. Matilla-Santander et al. [38] stated that insecure employment harms workers’ physical and mental health, which may be addressed in the future by equitable labour market improvements. Perna [39] underlines the need to regulate healthcare policies for precariously employed individuals in order for them to work healthily and live in dignity. Flandrick [40] analyzed various precarious employment characteristics that disproportionately affect women vs. men. Allowing for temporary employment, restricting women’s potential, rising inequality, financial inequalities, inadequate human rights protection, and inhumane working conditions are all challenges. Women’s labour market involvement is harmed by the aforementioned factors, leading to significant health repercussions.

The article "Do precarious female employment and political autonomy affect the under-5 mortality rate? Evidence from 166 countries" was retracted in 2024. Reasons: original data or images not available; unreliable results or conclusions; concerns about the data; concerns about the results or conclusions.

**Table 4:** Regression estimates.

Variables	Cross-sectional regression	Robust least squares regression	Quantile regression estimates
Constant	12.192*	14.459*	14.764*
Ln(FVE)	0.206*	0.164*	0.249**
ln(WPA)	-0.771*	-0.721*	-0.918*
ln(GDPPC)	-0.451*	-0.450*	-0.372*
Ln(IMUN)	-0.647*	-1.173*	-1.264*
**Statistical Tests**			
R^2^	0.793	0.723	0.583
Adjusted R^2^	0.788	0.716	0.573
Adjust Rw^2^	-----	0.843	-----
Rn-^2^	-----	647.133*	-----
F-statistics	154.383*	-----	-----
Quasi LR-statistic	-----	-----	289.567*

Note: U5MR shows an under-5 mortality rate, FVE shows female vulnerable employment, WPA shows women’s political autonomy, and GDPPC shows GDP per capita.

* shows 1% level of significance.

Additionally, the data reveal that women’s political autonomy and per capita income have a beneficial effect on achieving sustainable healthcare outcomes, as seen by a decrease in under-5 death rates across all countries examined. There is a negative association between sustained economic growth and decreased under-5 mortality rates in all three regression estimators. In light of the data, it seems that women’s engagement in economic and political activities benefits the long-term sustainability of health care. Women can better protect fundamental human rights, such as access to education and healthcare benefits since they possess more political savvy and economic means. Women may also participate in economic and commercial activities due to economic progress, which allows them to dedicate a greater share of their money to elementary education and women’s healthcare. Prior research confirms the aforementioned results, arguing that increasing funding for women’s empowerment has resulted in better health outcomes for women. According to Samanta [41], educated and mature women benefited from society’s health benefits by keeping their empowerment status, even though their empowerment was dependent on family support. Gammage et al. [42] conducted a critical analysis of the household and labour force surveys. They emphasised the importance of gathering additional critical data to reach definitive conclusions about women’s empowerment and access to reproductive healthcare. Women who are educated and engage in fair labour market reforms help women achieve autonomy, resulting in global healthcare advantages. According to Smith et al. [43], various issues impeded female empowerment and access to healthcare advancements, including gender inequality, racism, high healthcare expenses, and a lack of healthcare insurance services.

The article "Do precarious female employment and political autonomy affect the under-5 mortality rate? Evidence from 166 countries" was retracted in 2024. Reasons: original data or images not available; unreliable results or conclusions; concerns about the data; concerns about the results or conclusions.

Although all three regressions revealed a negative relationship between immunization rate and under-5 mortality rate, the quantile regression and robust least squares regression estimates revealed a more elastic relationship. In contrast, the cross-sectional estimates revealed a less elastic relationship. Consequently, increased vaccination coverage seems to reduce the risk of under-5 death rates. Numerous previous research has demonstrated the importance of increasing child vaccination coverage, which contributes to the worldwide reduction of health-related suffering. Patel et al. [44] emphasized the need to increase childhood vaccination to minimize morbidity and mortality. Maternal education is a critical aspect of increasing vaccination coverage. Hu et al. [45] proposed that increasing the vaccination worker-to-patient ratio might improve vaccine coverage and availability. Apart from vaccine assistance, governments and quasi-governmental organizations should priorities workforce development to boost kid vaccination rates. Allan et al. [46] discovered that a lower rate of complete immunization is associated with various characteristics, including children born at home, children born in rural regions, children born in disadvantaged households, and children born in higher birth positions. A component of project management will be devoted to identifying and vaccinating these under-vaccinated children to assist in the reduction of childhood vaccination inequities.

The diagnostic tests in Table 5 demonstrate that the regression estimates are devoid of serial correlation and homoscedasticity, suggesting that the regression estimates are normal.

**Table 5:** Diagnostic testing.

Variables	Variance Inflation Factor (VIF)	Diagnostic Testing	Estimated value	Probability value
ln(FVE)	2.790	J.B. Test	1.346^a^	0.509
ln(WPA)	1.292	LM (1) Test	3.593^a^	0.059
ln(GDPPC)	3.055	Heteroskedasticity Test	1.785^a^	0.152
ln(IMUN)	1.193	Ramsey RESET Test	0.632^a^	0.527
Quantile slope equality by Wald Test	8.028			
	(0.430)			
Symmetric Quantiles by Wald Test	4.010			
	(0.547)			

Note: J.B. shows Jarque Berra, LM shows Lagrange multiplier, FVE shows female vulnerable employment, WPA shows women’s political autonomy, GDPPC shows GDP per capita, and IMUN shows immunization coverage.^a^ estimates excluding a variable. Small bracket shows probability value.

The article "Do precarious female employment and political autonomy affect the under-5 mortality rate? Evidence from 166 countries" was retracted in 2024. Reasons: original data or images not available; unreliable results or conclusions; concerns about the data; concerns about the results or conclusions.

Additionally, Table 5 demonstrates no issue with multicollinearity since the VIF value is less than the threshold value of 10. The Wald test defined a temporal period, demonstrating that quantile regressions are stable in terms of quantile slope equality and symmetric quantile values. The results of the model stability tests indicate that the CUSUM and CUSUM square findings are statistically significant at a 95% confidence level; hence, the estimated model is stable over time (see Fig 4).

**Fig 4:** CUSUM and CUSUM square test estimates. Source: Author’s estimates.

The estimations in Table 6 reveal that GDP per capita will likely inflict larger variance error shocks on under-5 mortalities, with a shift of 0.652 percent in percentage terms. Following that, it is anticipated that women’s political autonomy and vulnerable female employment will grow by 0.302 percent and 0.212 percent, respectively, during the next decade. GDP per capita will continue to grow at a steady rate of 0.515 percent on average between 2023 and 2031. On the other side, it is expected that women’s political autonomy will increase from 0.272 percent in 2024 to 0.302 percent in 2031. Finally, it is expected that vulnerable female employment and vaccine coverage will increase from 0.206 percent and 0.045 percent in 2024 to 0.212 percent and 0.060 percent in 2031, respectively. The shocks are anticipated to have a stronger effect on the under-5 mortality rate, which is projected to decrease from 99.483 percent in 2023 to 98.771 percent in 2031.

**Table 6:** Variance decomposition of U5MR.

Years	S.E.	U5MR	FVE	WPA	GDPPC	IMUN
2022	28.50917	100	0	0	0	0
2023	28.75270	99.44340	3.43E-06	0.000662	0.515463	0.040469
2024	28.93693	98.83483	0.206975	0.272168	0.640773	0.045254
2025	28.94889	98.79288	0.207062	0.296460	0.646339	0.057255
2026	28.95243	98.77678	0.212862	0.301204	0.651743	0.057409
2027	28.95317	98.77179	0.212946	0.302761	0.651878	0.060628
2028	28.95324	98.77150	0.212981	0.302767	0.652116	0.060632
2029	28.95329	98.77123	0.212991	0.302800	0.652213	0.060770
2030	28.95329	98.77121	0.212991	0.302806	0.652219	0.060777
2031	28.95329	98.77120	0.212991	0.302806	0.652226	0.060777

Note: U5MR shows an under-5 mortality rate, FVE shows female vulnerable employment, WPA shows women’s political autonomy, GDPPC shows GDP per capita, and IMUN shows immunization coverage.

The article "Do precarious female employment and political autonomy affect the under-5 mortality rate? Evidence from 166 countries" was retracted in 2024. Reasons: original data or images not available; unreliable results or conclusions; concerns about the data; concerns about the results or conclusions.

The VDA projections are intended to help develop long-term, sustainable economic strategies for reducing child mortality under the age of five. Economic growth, according to estimates, will have a significant influence on the healthcare sustainability agenda in the following years. Increased funding for under-5 mortality reduction will contribute to the accomplishment of the United Nations Sustainable Development Goal #3. Women’s potential can be unleashed to improve their lives and lift themselves out of poverty and despair. Women who are empowered not only provide for their families but also have no problem acquiring healthcare benefits. To help women achieve the United Nations Sustainable Development Goals 5 and 8 in the context of precarious employment, labour reforms such as wage equity and equitable access to economic resources are necessary.

## 4. Discussion

The following key findings have been merged with the stated regression statistics, which have been discussed accordingly, i.e.,

- Maternal education may help lower infant mortality. The role of women n healthcare reproductive decisions should be strengthened by removing institutional and cultural barriers to reduce infant mortality [47].
- Family planning and prenatal care utilization were linked to higher levels of education, paid work, press coverage, and familial, economic status for women. Women’s autonomy may assist achieve gender equality and better usage of health care [48].
- Vaccination is one of the most effective strategies of illness prevention when fully covered. Lack of tetanus vaccination after birth was associated with lower socioeconomic status and fewer prenatal visits. These insights may help customize and execute the expanded immunization programme [49].
- Achieving regional and global vaccination objectives is typically difficult due to disparities in coverage. Assuring that all children have equal access to education, decision-making, and antenatal and postnatal care will help to improve full immunization coverage rates in low-performing areas [50].
- The national consensus on childhood immunization has helped reduce child mortality. One of the UN’s Sustainable Development Goals aims to decrease infant mortality to 25 per 1000 live births. It represented the child’s immunization status. Vaccination coverage was higher among children whose mothers were concerned about healthcare. Economic independence is influenced by self-determination, independence, mobility, and attitudes toward intimate partner abuse. Increasing child vaccination coverage will need a coherent approach to healthcare for the poor. More influence over their children’s and personal health might enhance vaccination programmes [51].
- Infectious illness vaccination timing is essential. Mumps patients may infect more individuals compared to polio patients. Individual protection against disease outbreaks may be achieved through timely immunization. Strong political commitment is required for universal childhood vaccination coverage [52].
- To narrow the vaccination coverage gap, more and sustained immunization is necessary. Preventing measles outbreaks requires widespread vaccination. This infectious and potentially lethal infection should be prevented by creative approaches to allow purpose vaccination [53], and
- Maternal and infant mortality are critical factors of healthcare sustainability—the WHO emphasizes a functional health care system to decrease unnecessary fatalities. Early intervention necessitates low-cost children, and a lack of medical facilities, infrastructure, staff, and pharmaceuticals may be the cause. There are several expanding markets affected by this issue. This reduces infant and mother mortality [54].

The article "Do precarious female employment and political autonomy affect the under-5 mortality rate? Evidence from 166 countries" was retracted in 2024. Reasons: original data or images not available; unreliable results or conclusions; concerns about the data; concerns about the results or conclusions.

Children under the age of five are a significant concern for researchers and community health specialists and a key indication of how families, communities, and the globe as a whole are progressing. Macroeconomic and health care aims and ideals of a nation are reflected in its policies. Despite the efforts of the government and other organizations, the death rate for children under the age of five continues to rise. Early and effective intervention is needed to address the criteria for under-five mortality [55].

## 5. Conclusions and policy implications

The research explores a variety of variables affecting the death rate of children under the age of five in a diverse range of nations. This was done via four factors: precarious female employment, women’s political autonomy, per capita GDP, and vaccination coverage. The first two SDG-5 (gender equality) elements are linked to fair labour reforms across countries. The third aspect pertains to SDG-5 (gender equality), whereas the fourth pertains to SDG-3 (ensure healthy living). GDP per capita and vaccination coverage are employed as a control variable to examine each nation’s overall economic situation, therefore contributing to SDG-3 and SDG-5. The regression findings indicate that vulnerable female employment is declining, which affects the accomplishment of SDG-3 and -5. By contrast, women’s political autonomy and economic prosperity contribute to the attainment of the United Nations’ SDG-3 goal of lowering child mortality. Immunization coverage increases the survival rate of children under five in all nations. According to the VDA research, countries’ per capita income will influence the under-5 mortality rate over the next decade, followed by women’s political autonomy, vulnerable female employment, and vaccination rate.

The article "Do precarious female employment and political autonomy affect the under-5 mortality rate? Evidence from 166 countries" was retracted in 2024. Reasons: original data or images not available; unreliable results or conclusions; concerns about the data; concerns about the results or conclusions.

Women’s health insurance benefits, labour market changes, and job-restructuring mechanisms should be included in long-term sustainable healthcare policies in a globalized society committed to improving healthcare and lowering infant mortality rates. Gender equality can enable women to fulfill their full potential in all fields of endeavour. Contributions of women to socioeconomic and environmental development are likely to strengthen their domestic and professional situations. Women who are educated, competent, and aware of their rights have a greater chance of accessing healthcare services. Women have been pushed to the bottom of the socioeconomic ladder due to the growing disparity between males and women in terms of educational and healthcare attainment. A country’s long-term development is contingent upon intelligent and broad-based policies in their promotion of gender equality. Preserving women’s employment opportunities and improving the labour market is crucial for attaining women’s autonomy. Women’s political intelligence and analytical talents enable them to capture a larger share of the labour force participation rate, which is declining in many civilized world regions. Women confront several other challenges in a male-dominated culture that must address women’s participation in political decision-making, along with job insecurity and unequal pay rates. The proposed revisions are meant to empower and help women on their journey to a happy and healthy life. More focus and effort must be directed on establishing policies that empower women in order for women to advance in overall healthcare rankings, owing to significant healthcare problems and a high rate of under-5 mortality in many areas. Female workers are also confronted with job market shifts, which must complement feminist measures such as paid maternity leave and a safe and secure work environment. Increased investment in women and girls is critical to preventing violence against them and ensuring equitable access to healthcare.

The following study shortcomings should be addressed in further research: The research relies on cross-sectional data from 166 countries to reach its results; however, using panel data series across countries may strengthen the study’s policy implications and generalizability. The research is confined to the four significant antecedents, but it might be broadened by integrating other control variables or confounding variables that could modify the investigated connections. The research examined the intertemporal interactions between time-independent variables. In comparison, cause-effect correlations between variables may be examined to understand them further and establish their causes.

The article "Do precarious female employment and political autonomy affect the under-5 mortality rate? Evidence from 166 countries" was retracted in 2024. Reasons: original data or images not available; unreliable results or conclusions; concerns about the data; concerns about the results or conclusions.

## Supporting information

S1 Appendix (DOCX)
